# A Random Forest Method for Identifying the Effectiveness of Innovation Factor Allocation

**DOI:** 10.1155/2022/1135582

**Published:** 2022-03-17

**Authors:** Mo Xu, Yawei Qi, Changqi Tao, Shangfeng Zhang

**Affiliations:** ^1^School of Statistics and Mathematics, Zhejiang Gongshang University, Hangzhou 310018, China; ^2^Collaborative Innovation Center of Statistical Data Engineering Technology & Application, Zhejiang Gongshang University, Hangzhou 310018, China; ^3^School of Information Management, Jiangxi University of Finance and Economics, Nanchang 330013, China; ^4^School of Statistics, Jiangxi University of Finance and Economics, Nanchang 330013, China

## Abstract

This paper makes a new attempt to identify the effectiveness of innovation factor allocation with a random forest method. This method avoids the evaluation bias of the relative effectiveness caused by the noneffective selection of production frontier in the nonparametric DEA method. It does not refer to other optimal subjects but shifts the focus to the judgment of its own effectiveness. In addition, it also gets rid of the constraints of the model and variables in the parameter SFA method, ensuring the reliability of the measurement results by resampling thousands of times. The data is collected from 30 provinces in China from 2009 to 2018. The findings show the innovation factor allocation in more than half of the provinces is not fully effective. It indicates that how to make use of innovation factor inputs to achieve the actual innovation output higher than own optimal levels is currently still in a period of exploration in China. To further improve innovation factor allocation efficiency, it deeply analyzes the impacts of innovation factor inputs and finds out the important innovation factor inputs. Furthermore, this study presents the nonlinear characteristics and optimal combination of important innovation factor inputs. According to this, it offers the detailed suggestions about how to adjust current important innovation factor inputs for each province in order to greatly enhance the effectiveness of innovation factor allocation in the future.

## 1. Introduction

After the outbreak of the new crown pneumonia epidemic, the global supply chain is forced to terminate, international and domestic demand are blocked, the barriers to the flow of factors are strengthened, and the phenomenon of factor misplacement aggravates. And the five major technologies of big data, cloud computing, Internet of Things, blockchain, and artificial intelligence emerge contribute to the vigorous development of the real economy and bring the great value of the digital economy. As a basic resource in the digital economy, data factors promote the transformation and upgrading of other production factors. The optimization of the spatial layout of regional innovation factors is inseparable from the support and guidance of government policies. This not only reflects that new innovation factors such as data and institution have significantly affected the transformation of productivity and production relations, but also broadens the connotation scope of the original traditional innovation factors. In addition, the distribution of innovation factor inputs is uneven and innovation capability is generally low among provinces in China, while the calculation results of innovation efficiency are controversy. It is of great practical significance to identify the effectiveness of innovation factor allocation in each province under the new connotation of innovation factors. To this end, clarifying the multidimensional characteristics of innovation factors, selecting reliable measurement methods, and analyzing the current situation of innovation factor allocation in each province play a powerful role in stimulating the innovation factors potential and driving economic growth.

The existing literature measures the allocation efficiency of innovation factors roughly from the following three levels: First, different innovation inputs and innovation outputs. Duan et al. [1] construct a comprehensive index of innovation development from the three dimensions of innovation inputs, innovation organization, and innovation outputs. Dai et al. [2] use financial resources as scientific and technological financial inputs, and scientific and technological achievements as scientific and technological financial outputs. Tao and Peng [3] regard internal R&D expenditures and full-time equivalent of R&D personnel as technological innovation inputs, and the number of patent applications received, revenue from new product sales, and revenue from main operations as technological innovation outputs. Second, different innovation efficiency evaluation objects and various innovation efficiency measurement ways. Li et al. [4] decompose the innovation process into innovation development process and innovation transformation process and then calculate the innovation efficiency of 37 subsectors in China from 2004 to 2011. Wang and Lan [5] use the SFA model to estimate the innovation efficiency of China's A-share listed state-owned enterprises. Chen and Li [6] adopt a two-stage network DEA method to obtain the green innovation efficiency, green technology research and development efficiency, and green technology achievement conversion efficiency in China from 2003 to 2017. Third, measure the allocation efficiency by the factor allocation distortion. Dollar and Wei [7] find that the systematic distortion of capital allocation in China leads to uneven marginal returns across companies, regions, and departments. They point out that if capital can be allocated more effectively, it can lower capital intensity by 5% without sacrificing economic growth. Hsieh and Klenow [8] find that if capital and labor are redistributed so that the marginal output of China and India is equal to that of the United States, this will increase the total factor productivity of the manufacturing industries of the two countries, respectively, by 30%–50% and 40%–60%. Chen and Hu [9] show that resource misallocation leads to a gap of about 15% between actual output and optimal output in various subsectors of China's manufacturing industry.

Existing researches which discuss the allocation modes of innovative factors mainly can be divided into internal, external, and open innovation. Internal innovation means that the innovation subject relies on its own innovation factors to achieve innovative production. External innovation means that the innovation subject completes innovation activities with the help of external innovation factors. Open innovation means that the innovation subject breaks through its own innovation boundaries and coordinates internal and external innovation factors in the innovation process [10]. However, different ways of allocating innovation factors have different impacts on innovation performance. Hong and Shi [11] believe that independent R&D is significantly positively correlated with enterprise innovation performance. Chen and Hou [12] find that the influence of independent innovation on scientific and technological performance manifests a nonlinear threshold effect. Kafouros et al. [13] conclude that the impact of academic cooperation on the innovation performance in Chinese emerging market companies is significantly positive. Asimakopoulos et al. [14] point out that there is an inverted U-shaped relationship between external knowledge and enterprise innovation efficiency. Berchicci (2013) [10] believes that the inverted U-shaped relationship between external R&D activities and enterprise innovation performance is the function of the substitution effect of its own R&D capabilities. Nieves and Petra [15] find that internal and external knowledge have substitution effects within a certain threshold and have a negative impact on enterprise innovation performance. When the threshold is exceeded, it will turn into a complementary effect and has a positive impact on the enterprise innovation performance.

In summary, the definition of the connotation of innovation factors in the existing literature is mostly based on the traditional innovation factors such as labor, capital, and technology. But it lacks the content of new innovation factors such as data and institution. The existing literature ignores the theoretical basis and operation process behind the innovation factor allocation. The efficiency measurement of the innovation factor allocation in the existing literature is mostly by means of the parametric SFA and the nonparametric DEA. In addition, there are few studies on the evaluation of innovation factor allocation effectiveness. Adopting a more reliable method to identify the effectiveness of innovation factor allocation is helpful to evaluate the situation of innovation factor allocation more accurately. In view of this, the main contributions of this article are as follows: On the one hand, with the introduction of the data and institution innovation factors, we build the index of multidimensional innovation factor, which not only weighs the internal and external coordination of traditional innovation factor from the cost theory, but also considers the moderating effect of new innovation factor from the coupling theory. Based on this, a four-dimensional integrated indicator is formed including internal innovation factors, external innovation factors, institutional innovation factors, and data innovation factors and the allocation of innovation factor is evaluated on the input-output process of innovation factor. On the other hand, we make a new attempt to identify the effectiveness of innovation factor allocation by a random forest method that is different from the previously used. This method can not only get rid of constraints including the model setting form, the number of variables, and the correlation between variables in the parameter SFA method, but also avoid the evaluation bias of the relative effectiveness caused by the noneffective selection of production frontier in the nonparametric DEA method. It shifts the focus on its own efficiency, ensuring the reliability of the measurement by resampling thousands of times. The above aspects are the contribution of the theoretical level. Furthermore, in the aspect of practical level, we draw many different conclusions from existing studies, which find that the innovation factor allocation in more than half of the provinces is not fully effective, data innovation factor inputs especially data integration and data applications have the significant contribution to innovation output, the marginal impact characteristics of important innovation factor inputs are all nonlinear, and the gap between the current situation and the optimal combination of important innovation factor inputs in each province in China is obvious, etc.

The remaining structure of this paper is as follows: In Section 2, we present the definition and measurement method of innovation factor allocation. In Section 3, we identify the effectiveness of innovation factor allocation in each province in China and discuss the importance of innovation factor inputs. In Section 4, we determine the important innovation factor inputs, describe their nonlinear characteristics and optimal combination, and then point out the future adjustment direction of innovation factor inputs in each province in China. In Section 5, we offer the main conclusions and future research.

## 2. Innovative Factors: Definition, Indicator, and Measurement Method

### 2.1. Definition

#### 2.1.1. The Definition of Innovation Factors

Production factors are the objective basis of production activities, and factors affecting production activities all belong to the category of factors [16]. The narrow defining of production factors can be understood as the factors joining in the production process, while the broad defining of production factors should also include factors that reflect the output benefits of the production process. Schumpeter [17] defines innovation as introducing a new combination of production factors and production conditions into the production system that has never been before. Combining modern production conditions with organizational models, innovation can be understood as not only the realization of new products (services) or procedures, the improvement of original products (services) or procedures, but also the process of new products (services) or procedures that are about to or have been commercialized [18–20].

To sum up, this article defines innovation factors as production factors that participate in the innovation process, influence innovation performance, and reflect innovation achievements. They have the characteristics of increasing marginal returns, which include not only traditional innovation factors such as labor, capital, and technology, but also new innovation factors such as data and institution.

#### 2.1.2. The Definition of the Multidimensional Innovation Factor Allocation

The cost theory holds that the criterion for organizing economic activities is the minimization of internal production costs and external transaction costs. Drawing on Nieves and Petra (2014) [15], the innovation factors are divided into internal innovation factors and external innovation factors, the internal innovation factors are derived from the innovation subject itself, the external innovation factors are derived outside the innovation subject, and the internal and external innovation factors are mainly based on traditional innovation factors. On the one hand, the innovation subject relies on internal innovation human, material and financial resources, regards innovation as an internal control process, completes all innovation links and leaves innovation output within the subject. On the other hand, the innovation subject combines their own existing innovation foundations and regards innovation as a R&D outsourcing process. By contacting external innovation partners, they achieve technology cooperation, absorption, and acquisition of external innovation and enlarge enterprise innovation outputs. If the innovation subject is overconcentrated on internal innovation, it will cause problems such as excessive risk and knowledge spillover, while overreliance on external source innovation will bring about problems such as rising negotiation costs and loss of initiative. Therefore, the innovation subject needs to effectively coordinate internal and external innovation factors to minimize the total cost of innovation activities.

The coupling theory states integrating the coordination channels of internal and external traditional innovation factors, enhancing the coupling viscosity of internal and external traditional innovation factors, and reducing the misallocation of internal and external traditional innovation factors, which require both the participation of innovation subjects themselves and innovation assistance from forces other than the subjects. We refer to analysis of Berchicci [10]. On the one hand, the government-led institutional innovation factors regulate the depth of internal and external innovation factors coordination, integration, and fit by intellectual property protection, financial education support, free trade in goods, market transaction quotas, financial development scale, and industrial pollution control. On the other hand, data innovation factors led by intermediaries regulate the breadth of internal and external innovation factors synergy, integration and adaptation by data production level, data transmission speed, data user groups, data application scope, data sharing degree, and data integration capabilities. Institution and data innovation factors play the regulatory role of institutions and information (intrinsic nature of data) on internal and external innovation factors, thereby forming a multidimensional integrated indicator of internal innovation factors, external innovation factors, institutional innovation factors, and data innovation factors.

Based on the above analysis, this article draws the definition of the multidimensional innovation factor allocation. The cost theory synergizes internal and external innovation factors. The measurement indicator of internal innovation factors can be from the three aspects of internal innovation human resources, material resources, and financial resources. The measurement indicator of external innovation factors can be from three aspects such as external innovation technologies cooperation, absorption, and acquisition. The regulation role of institution and data innovation factors depends on coupling theory. Institution innovation factor measurement indicator can be from six aspects including property rights protection, education support, trade freedom, trading markets, financial development, and pollution control. Data innovation factor measurement indicator can be from six aspects including data generation, transmission, use, application, sharing, and integration.

### 2.2. Indicator

#### 2.2.1. Indicator Composition

This paper is based on the definition of innovation factors allocation, the operability of indicators, and the availability of data. Combining with the research of Tao and Xu [21], we select the specific quantitative indicator. The internal innovation human resources, financial resources, and material resources in the internal innovation factors are, respectively, measured from the full-time equivalent of R&D personnel, internal R&D expenditures, and the number of R&D organizations. The external innovation technology cooperation, absorption, and acquisition in external innovation factors are, respectively, measured from external R&D expenditures, foreign direct investment, and high-tech product imports. Property rights protection, education support, trade freedom, trading market, financial development, and pollution control in the institution innovation factors are, respectively, measured from the total number of patent enforcement cases, financial education subsidies, total regional goods exports, technology market turnover, deposits and loans of financial institutions, and industrial pollution control investment. The data generation, transmission, use, application, sharing, and integration in the data innovation factors are, respectively, measured from the number of Internet pages, Internet broadband access ports, Internet users, total software services, total post and telecommunications services, and the number of robots owned. Taking the above four dimensions of internal, external, institution, and data innovation factors as innovation inputs, and taking per capita sales income of new products as innovation output, we evaluate China's innovation factors allocation efficiency.

#### 2.2.2. Variables and Data

This paper is based on the panel data of 30 provinces in China from 2009 to 2018 (except Tibet). The data are extracted from China Statistical Yearbook on Science and Technology, China Statistical Yearbook, China Internet Development Report, China Information Yearbook, and International Federation of Robotics. The acquisition of the variables and the processing of the data are performed as follows: Regarding the matches and fillings of the data, the first is the number of robots owned in China based on the industrial output value of the main applications of industrial robots in each province. The second is filling the missing data of provinces according to the difference between the national total and existing provinces total. In addition, with regard to the methods of the processing of the data, firstly, exchange rate adjustments are converted by the ratio of RMB to USD. Secondly, the price adjustment refers to the price index formula of Zhu and Xu [22]. The fixed asset investment index and the consumer price index are, respectively, assigned weights of 0.45 and 0.55. Regarding the year 2009 as the price base period, convert the nominal values into actual values. Thirdly, using the method of BEA for stock adjustment, based on the annual investment flow after price adjustments *E*_*t*_, we calculate the average annual growth rate *g*_*k*_. Then, considering amortization of intangible assets for at least 10 years, and referring to Wang and Gao [23], set the residual value rate *d*_*T*_ to 10% and get the depreciation rate *δ*=1 − (*d*_*T*_)^1/*T*^=0.2057. Lastly, the annual capital stock is based on *K*_0_=[*E*_1_(1 − *δ*/2)]/[*g*_*k*_+*δ*] and *K*_*t*_=(1 − *δ*)*K*_*t*−1_+(1 − *δ*/2)*E*_*t*_. The above contents are detailed in Table 1.

### 2.3. A Random Forest Method

The existing researches of measuring efficiency mainly use nonparameter DEA method and parameter SFA method. The DEA method is used to evaluate relative efficiency by constructing the optimal production frontier. On the one hand, it refers to other effective subjects instead of its own optimum, which is difficult to purposely offer the adjustment direction according to itself current inputs. On the other hand, it may occur efficiency measurement bias if the optimal production frontier is selected mistakenly. In addition, the SFA method measures efficiency by determining the form of model and the number of variables in advance. It means the differences of the form of model and the number of variables lead to the different measurement results. Meanwhile, the collinearity between variables in the model also causes biased efficiency measurement. Compared with DEA and SFA, the random forest method not only gets rid of constraints including the form of model, the number of variables, and the correlation between variables, but also ensures the reliability of measurement by resampling thousands of times. With reference to Ouyang and Chen [24], the prediction of output can be regarded as the maximum output achieved under the full utilization of inputs by the random forest method. According to this, we can calculate own optimal output in terms of current inputs and then identify effectiveness by the ration of actual output to optimal output. It does not refer to other optimal subjects but shifts the focus to the judgment of its own effectiveness. Moreover, it gets the contribution rankings of various inputs to outputs from large to small based on the principle of minimum sum of squares of residuals. We further get the marginal impact characteristics of inputs and find out the optimal combination of inputs and thus put forward the further adjustment direction depending on own current situation of inputs. The introduction of random forest method is below in detail.

A random forest method is an ensemble learning method. This method uses resampling to randomly select sample data and sample characteristics to establish multiple regression numbers, and the mean value of the output results of multiple regression trees is used as the final prediction result. Based on the data of each input, this paper predicts the results of each output according to the random forest method. The detailed steps are as follows:

(i) Suppose there are samples {*y*_*i*_, *c*_*i*1_, ..., *c*_*iK*_}_*i*=1_^*N*^, *N* and *K*, respectively, represent total number of samples and features, *y*_*i*_ is the individual *i* output, and *c*_*i*1_, ..., *c*_*ik*_ is the individual *i* input. Based on this, samples are drawn randomly with replacement.
(ii) Construct a regression tree with features *m* selected from the sample, and perform feature splitting according to the principle of the minimum sum of squared residuals. Specifically for the input indicator *c*_*k*_, the critical point at which the optimal threshold is known is *d* (the determination of *d* also adopts the principle of minimum sum of squares of residuals). Then according to the sample size of the left and right sides of the critical points *T*_*U*1_ and *T*_*U*2_, we, respectively, get the sample of *U*1 and *U*2:
  (1) $$\begin{array}{c} U1\left(k,d\right)={\left\{y_{i},c_{i1},...,c_{iK}/c_{k}\leq d\right\}}_{i=1}^{T_{U1}},\;U2\left(k,d\right)={\left\{y_{i},c_{i1},...,c_{iK}/c_{k}>d\right\}}_{i=1}^{T_{U2}}. \end{array}$$

From this, the average value of the output results of each sample can be obtained:

(2) $$\begin{array}{c} {\bar{y}}_{U1}=mean\left(y_{i}/y_{i}\subseteq U1\right),\;{\bar{y}}_{U2}=mean\left(y_{i}/y_{i}\subseteq U2\right). \end{array}$$

The selection of the initial split node *c*_*k*_ of the regression tree is based on the following formula:

(3) $$\begin{array}{c} \underset{C_{k}}{\min}\left[\min\sum_{i=1}^{T_{U1}}{\left(y_{i}-{\bar{y}}_{U1}\right)}^{2}+\min\sum_{i=1}^{T_{U2}}{\left(y_{i}-{\bar{y}}_{U2}\right)}^{2}\right]. \end{array}$$

- The selection of the remaining nodes of the regression tree is repeated based on step (ii). The prepruning rule is set to include at least 5 sample points for each node. When the rules are met, the regression tree immediately stops splitting.
- The loop steps (i)-(iii) form a large number of regression trees, and the average value of the above regression tree results is used as the final prediction of the output results.

In addition to regression analysis, the random forest method can also evaluate the importance of each input and its marginal influence on the output. The nodes of the regression tree are arranged from top to bottom according to the contribution of each input to the reduction of the residual sum of squares of the output. The top is the input with the largest contribution, and the bottom is the input with the least contribution. According to this, the importance of each input can be obtained. By sorting the importance of input, we can get the important order of input. The marginal effect is mainly used to measure the impact of a single input change on the output, which can be defined as

(4) $$\begin{array}{c} \bar{f}\left(c_{k}\right)=\frac{1}{N}\sum_{i=1}^{N}f\left(c_{i1},...,c_{k},...,c_{iK}\right). \end{array}$$

In equation (4), *f*(*c*_*i*1_, ..., *c*_*k*_, ..., *c*_*iK*_) is the prediction result of the random forest model *f*(·) when {*c*_*i*1_, ..., *c*_*k*_, ..., *c*_*iK*_}_*i*=1_^*N*^ is known. $\bar{f}\left(c_{k}\right)$ is the mean of the predicted results for all samples. Traverse all possible values *c*_*k*_ to get the corresponding result $\bar{f}\left(c_{k}\right)$. This draws a trend graph $\bar{f}\left(c_{k}\right)$ about *c*_*k*_ and visualizes the influence path of the input *c*_*k*_ on the mean value of output $\bar{f}\left(c_{k}\right)$.

## 3. Innovation Factors: Allocation Effectiveness and Importance Degree

### 3.1. Effectiveness Identification

We use random forest method, the algorithm is run 1000 times, and the average value of 1000 times is regarded as the final prediction of innovation output. Based on the above analysis, it is also the optimal innovation output achieved by innovation factor inputs. Then we get the ration of actual output to optimal output, which is the allocation efficiency of innovation factors from 30 provinces in China from 2009 to 2018. Based on this, we identify the effectiveness of innovation factor allocation for each province in China and offer the corresponding schematic graph shown in Figure 1.

In Figure 1, the black solid dots indicate that the province's actual innovation output exceeds its own optimal output, realizing the effective allocation of innovation factors, while the gray solid dots indicate that the province's actual innovation output is lower than its own optimal output. The effective allocation of innovation factors has not been completed. According to the allocation of innovation factors in each province from 2009 to 2018, each province is divided into the following three types: one is fully effective, and the province achieves an effective allocation of innovation factors during the entire sample period; the second is not fully effective, and the province only achieves the effective allocation of innovation factors in a part of the sample period; the third is totally ineffective, and the province does not meet the requirements of the effective allocation of innovation factors during the full sample period.

As can be seen from Figure 1, the provinces with innovation factor allocation fully effective are Tianjin, Shanxi, Shanghai, Zhejiang, Hubei, Hunan, Chongqing, and Ningxia. The above provinces can not only effectively coordinate internal and external innovation factors during the entire sample period, but also give full play to the coupling role of institution and data innovation factors, organically integrate the four-dimensional innovation factors into one, and obtain innovation output that exceeds its own best state. Although Chongqing and Ningxia are located in the relatively backward western regions, there is a certain gap in the innovation factor inputs compared with the developed regions, and the optimal output that can be achieved by the current innovation factor inputs is relatively low, so the actual output of the two provinces reaching the optimal level is also relatively easy. The provinces where the allocation of innovation factors is not fully effective are Beijing, Inner Mongolia, Liaoning, Jilin, Jiangsu, Anhui, Fujian, Jiangxi, Shandong, Guangdong, Guangxi, Gansu, Qinghai, and Xinjiang. In the abovementioned provinces, the innovation output obtained by the innovation factor inputs in only some years is higher than its own optimal level. Although Beijing, Jiangsu, Fujian, Shandong, and Guangdong are located in eastern regions with superior innovation conditions and abundant innovation resources, their innovation factor inputs are relatively more, and the optimal output that can be achieved by relying on their existing innovation factor inputs is also relatively high. The actual output beyond its own optimal level is also relatively difficult. The provinces where the allocation of innovation factors is totally ineffective are Hebei, Heilongjiang, Henan, Hainan, Sichuan, Guizhou, Yunnan, and Shaanxi. The actual output of the above eight provinces during the entire sample period was lower than their optimal level. Although Hebei is located in the economically developed eastern region, the relatively high innovation factor inputs have caused structural imbalance, and it is difficult to fully release the efficacy of innovation factor inputs.

### 3.2. Importance Judgment

From the foregoing, the random forest method can get the importance of the innovation factor inputs according to the contribution to the reduction of the square of the residual of the innovation output. It puts the most important innovation factor input at the top of the tree and the least important innovation factor input at the bottom of the tree. Therefore, the higher the innovation factor input located at the level of the tree, the greater the contribution to the innovation output. According to the importance of the innovation factor inputs from 2009 to 2018 (see Table 2), this paper draws a grid graph and a boxplot graph (see Figures 2 and 3). The grid graph reflects the contribution degree, the changing trend, and the abnormal time point. The larger the grid area, the greater the importance. The boxplot presents the average contribution and scatter degree. Based on the above analysis, it provides clear direction for improving the effectiveness of innovation factor allocation.

In Table 2 and Figure 2, it can be seen that the contribution of data application is the most prominent in 2009 and 2010, the contribution of external innovation technology absorption is the most significant in 2013 and 2018, and the performance of data integration is the most eye-catching in the remaining years, which show that the data application, external innovation technologies absorption, and data integration have significant impacts on the innovation output during the entire sample period. In addition, the number when the input of innovation factors contributes the most value itself is as follows. First, the number topping the list in 2018 is five, respectively, including internal innovation human resources, external innovation technology cooperation, external innovation technology absorption, financial development, and pollution control. Second, the number in 2010 is four, respectively, including external innovation technology acquisition, education support, trading market, and data application. Third, the number in 2009 and 2016 is three, which, respectively, include property rights protection, data transmission and data use in 2009, and internal innovation financial resources, internal innovation material resources, and data integration in 2016. Forth, the number in 2013 is two, respectively, including trade freedom and data sharing, the input in 2015 is data generation, and there is none in 2011, 2012, 2014, and 2017. This shows that the input structure of innovation factors in 2018 is more reasonable than other years, it gives full play to the advantages of innovation factor inputs, and there is the most innovation factor input contributing its greatest impact.

In Table 2 and Figure 3, the average contribution of innovation factor inputs during the entire sample period is ranked from large to small, followed by data integration, data application, external innovation technology absorption, internal innovation material resources, external innovation technology acquisition, financial development, internal innovation human resources, trade freedom, internal innovation financial resources, data generation, external innovation technology cooperation, trading market, data transmission, data sharing, data use, property rights protection, pollution control, and education support. The ranking top two belong to data innovation factors. It confirms not only the importance of the data innovation factor inputs, but also the data integration measured by the number of robots owned and the data application measured by the total amount of software business, which implies artificial intelligence and advanced manufacturing playing the important role within reforming the synergy of internal and external innovation factors and promoting the acceleration of innovation output. Data innovation factors have the characteristic of strong integration. They can overcome the limitations of time and space, which is conducive to the optimization and upgrading of internal and external innovation factors and the complementary advantages between internal and external innovation factors, which greatly promotes the improvement of innovation output. Internal innovation human resources, internal innovation financial resources, external innovation technology absorption, education support, pollution control, and data transmission all have outliers. Five have large outliers which all appear at the largest time point of its own contribution, and three appeared in 2018. It not only illustrates the relatively reasonable input structure of innovation factors in 2018, but also implies that the overall input structure of innovation factors in China is undergoing continuous adjustment and improvement.

## 4. Innovation Factors: Marginal Effects and Input Choices

### 4.1. Marginal Effect Trend

The above discusses the importance of each innovation factor input to the innovation output under the existing innovation factor inputs combination, which is the static analysis of the impact on the innovation output. If the innovation factor input has a significant impact on innovation output, will it continue to increase inputs or be subject to threshold constraints? The answer to this question requires us to give the dynamic changes in the marginal effect trend of innovation factor input.

Based on the importance ranking of innovation factor inputs, the top eight cumulative impacts exceeding 60% of the total impact are regarded as important innovation factor inputs, followed by data integration, data application, external innovation technology absorption, internal innovation material resources, external innovation technology acquisition, financial development, internal innovation human resources, and trade freedom. At the same time, it is found that the above inputs are evenly distributed in the internal, external, institution, and data innovation factors. In order to obtain the time changing trend of the marginal effects of each important innovation factor, the marginal effect graph of each important innovation factor input is given in the order of the abovementioned four-dimensional innovation factors (see Figure 4). We select 2009 (dotted line type), 2012 (lower solid line), 2015 (dashed line), and 2018 (higher solid line) for describing in detail.

There are three key boundary points in the marginal effect trend graph in Figure 4, which are two turning points (indicated by ×) and the maximum slope point (indicated by *∗*). Before the first turning point is the initial stage of innovation factor input impact, and the marginal impact on innovation output is relatively flat. The first turning point to the maximum slope point is the marginal impact on innovation output from the increasing to the maximum. The stage between the maximum slope point and the second turning point is the marginal incremental impact of the innovation factor input fallen to the suspended. The second turning point is the innovation factor input required for maximum innovation output. The marginal impact of increasing the innovation factor input on innovation output is almost zero after the second turning point. It can be concluded that the optimal innovation factor is the amount of innovation factor input required when the innovation output reaches its maximum output. If all the important innovation factor inputs in a province have exceeded the second turning point, then the province's important innovation factor investment portfolio is the best. Based on this, we give the key boundary points of the marginal effect of important innovation factor inputs in 2009, 2012, 2015, and 2018 (see Table 3).

Combining the time trend of the marginal effects of important innovation factors, we find that the impact on innovation output is nonlinear in whole process. In addition, the positions of the first turning point, the maximum slope point, and the second turning point are not exactly the same in 2009, 2012, 2015, and 2018. It can be seen that the demand for important innovation factor inputs in different periods is somewhat different. Details are as follows: Firstly, the first turning point of internal innovation human resources, financial development, and data integration between 2009 and 2015 is relatively closer. The distance of the first turning point in internal innovation material resources, external innovation technology acquisition, and data application between 2012 and 2015 is the shortest. At the same time, except for trade freedom, the first turning point of the other important innovation factor inputs in 2018 appears later than the other years. It shows that the amount of the important innovation factor inputs required at the starting point of increasing marginal effects in 2009, 2012, and 2015 is relatively stable, while the amount of the important innovation factor inputs required in 2018 is higher than that in 2009, 2012, and 2015. Secondly, the distance of all important factor inputs between the first turning point and the maximum slope point in 2018 is smaller than in 2009, 2012, and 2015. It indicates that, compared with other years, the important innovation factor inputs have the certain foundation and do not have a relatively long period of marginal effect growth in turn in 2018. Thirdly, the second turning point of internal innovation human resources in 2018 appears earlier than in 2009, 2012, and 2015, while the second turning point of the other important innovation factors in 2018 appears later than in 2009, 2012, and 2015. It indicates that, comparing 2018 with the other years, the demand for internal innovation human resources is relatively small, and the demand for other important innovation factors is greater in the optimal innovation factor inputs required to achieve the maximum innovation output.

### 4.2. Inputs Selection Analysis

The ranking top eight of the innovation factor inputs' importance in 2012 and 2018 are consistent with the result of the average contribution ranking in Table 2. Therefore, the input of important innovation factors in each province in 2012 and 2018 is carried out by grouping accordingly. It can not only analyze the time changes of important innovation factor inputs, but also propose future adjustment direction based on the current innovation factor inputs in each province.

According to the grouping of important innovation factor inputs in each province in 2012 and 2018 (see Table 4), combined with the marginal effect graph of important innovation factor inputs in 2012 and 2018 (see Figures 4(a)–4(h), respectively, corresponding to the lower and the higher solid line), the following important features are found: Firstly, part of important innovation factor inputs in some provinces have not exceeded the critical value of the first turning point. That means these important innovation factor inputs have not yet reached the starting point of increasing marginal effects. Secondly, all important innovation factor inputs in some provinces are between the first turning point and the second turning point. That indicates all important innovation factor inputs are in the stage where their marginal effect increases to the maximum and then to the gradual decline. Thirdly, part of important innovation factor inputs in some provinces have reached the second turning point threshold value, which means that these important innovation factors have completed the optimal inputs. Fourthly, all important innovation factor inputs in some provinces exceed the second turning point threshold value, which indicates that all important innovation factor inputs meet the optimal portfolio requirements. Based on the above four important characteristics, we classify the input of important innovation factors in each province in 2012 and 2018, analyze the characteristics of changes in the important innovation factor inputs, and propose future innovation development policies.

Based on the summary of important innovation factor inputs grouping characteristics in each province in 2012 and 2018 (see Table 5), the changes in the following grouping characteristics of each province are obtained: Firstly, the important innovation factor inputs in some provinces in 2012 and 2018 have always maintained the characteristics (a), such as Qinghai and Ningxia. Although Ningxia shows the innovation factor allocation is effective in 2012 and 2018, the optimal innovation output achieved is low due to its existing innovation factor inputs. It implies that the above provinces need to significantly increase the important innovation factor inputs, which can not only increase the actual innovation output, but also raise the optimal output threshold standard. Secondly, the important innovation factor inputs in some provinces in 2012 and 2018 remain at the characteristic (b), such as Tianjin, Hebei, Liaoning, Jilin, Anhui, Henan, Hunan, and Chongqing. The above provinces may refer to the contribution ranking of important innovation factor inputs and determine the appropriate direction for the increase in the important innovation factor inputs. There are also some provinces where the important innovation factor inputs have dropped from the characteristics (b) in 2012 to the characteristics (a) in 2018, such as Shanxi, Inner Mongolia, Heilongjiang, Jiangxi, Guangxi, Hainan, Guizhou, Yunnan, Gansu, and Xinjiang. The above provinces input less in data applications. The contribution of data application input is among the best. Increasing the inputs of data application can not only make the provinces get rid of the characteristics (a), but also promote the improvement of innovation output. There are also some provinces where the investment in important innovation factors has risen from the characteristic (b) in 2012 to the characteristic (c) in 2018, such as Fujian, Hubei, Sichuan, and Shaanxi. The grouping characteristics have been upgraded, and the above provinces need to continue to maintain this situation, or they can increase investment in innovation factors which have a large gap such as trade freedom and other factors. Thirdly, the input of important innovation factors in some provinces in 2012 and 2018 has always remained at the characteristic (c), such as Beijing, Shanghai, Zhejiang, and Shandong. The above provinces may be based on the gap of some important innovation factors between current and optimal inputs, combined with the contribution of important innovation factor inputs, giving priority to the important innovation factors with small gaps and large contributions. Fourthly, the inputs of important innovation factors in Guangdong in 2012 and 2018 have met the requirements of characteristics (d). It means that Guangdong has realized the effective allocation of innovation factors in 2018. If they want to improve the optimal innovation output standard, it is more difficult to start from the input end of innovation factors. It may be achieved by changing the existing innovation development patterns. The important innovation factor inputs in Jiangsu Province have declined from the characteristics (d) in 2012 to the characteristics (c) in 2018. Jiangsu Province may continue to increase inputs in financial development and data applications in the future.

## 5. Conclusions and Future Research

Innovation is the driving force of economic development, and effectively measuring the allocation of innovation factors is conducive to better playing the role of innovation. We use the random forest method to identify the effectiveness of innovation factor allocation in 30 provinces in China from 2009 to 2018 and explore the importance of the innovation factor inputs' contribution in the entire sample period and its own maximum contribution timing. Then we further grasp the marginal effect characteristics of important innovation factor inputs, catch the time changes of its key boundary points, analyze the actual inputs of each province based on the optimal combination of important innovation factor inputs, and finally propose future adjustment directions. The specific conclusions reached are as follows.

First, more than half of the provinces is not fully effective in the innovation factor allocation. How to rely on internal and external innovation factors and make use of institution and data innovation factors to achieve the actual innovation output higher than their own optimal levels is still in a period of exploration and adjustment. Second, from the perspective of the importance of innovation factor inputs, data innovation factors especially data integration and data applications have contributed significantly, which reflects the important impact of data innovation factors on innovation output. From the view of the maximum contribution time of innovation factor input, the most innovation factor inputs contribute its own maximum value in 2018, suggesting that the structure of China's innovation factor input has an overall upward development trend. Third, the marginal effects of important innovation factor inputs are nonlinear, and the positions of the first turning point, the maximum slope point, and the second turning point of the marginal effect of important innovation factor inputs in different periods are different, indicating that the marginal effect of important innovation factor inputs on innovation output is not always the same. Based on this, we find out the optimal combination of important innovation factor inputs. Fourth, Guangdong Province has achieved the optimal combination of important innovation factor inputs or can change the existing innovation development pattern, while the remaining provinces have not yet reached the optimal factor input requirements and need to adjust the inputs to improve the current innovation choice.

Based on the above conclusions, the following policy implications can be obtained. Firstly is improving the effectiveness of the innovation factor allocation further. We not only need to pay attention to the coordination of internal and external innovation factors, but also focus on the coupling of institution and data innovation factors. Secondly is giving full play to the potential of data innovation factors, especially data application and data integration: Developed provinces may be able to make further development, while backward provinces may be able to achieve curve overtaking. Thirdly is grasping the marginal effects of important innovation factor inputs, and making good use of the impact trend of the important innovation factor inputs. Fourth, each province makes appropriate innovation development policies based on local conditions and rationally adjusts the current innovation factor inputs selection according to the optimal combination.

Needless to say, this paper has some limitations, which are also the basis of future research in this paper. Firstly, when evaluating the effectiveness of innovation factors allocation, this paper takes internal innovation factors, external innovation factors, institutional innovation factors, and data innovation factors as innovation factor inputs, and per capita new product sales revenue as innovation output. Except for per capita new product sales revenue, it can also be measured by indicators such as per capita gross national product in the evaluation of innovation output. Therefore, it is necessary to add other variables that can measure innovation output to identify the effectiveness of innovation factor allocation in further research, so as to more comprehensively show the allocation situation of innovation factors in various provinces in China.

Secondly, this paper takes China's provinces as the research object and evaluates the innovation factor allocation from the macrolevel. In addition, it also has practical significance of evaluating the innovation factor allocation from the meso- and microlevels. Therefore, it is necessary to analyze the innovation factor allocation from the industry level and the enterprise level and further explore the future adjustment direction of the innovation factor allocation at the meso- and microlevels.

Finally, when analyzing the impact of innovation factor input, this paper focuses on the marginal effect trend and key boundary points of important innovation factor input but does not show the impact of remaining innovation factor input on innovation output. Although the impact of this part of innovation factor inputs is not significant, they also make the marginal contributions to innovation output. In the future, we may further explore the marginal effect characteristics and key boundary points of such innovation factor inputs. It may draw other important conclusions.

## Figures and Tables

**Figure 1:** Effectiveness of innovation factor allocation.

**Figure 2:** Grid graph of innovation factor inputs importance.

**Figure 3:** Boxplot of innovation factor inputs importance.

**Figure 4:** Marginal effect trend of important innovation factor inputs. (a) Internal innovation human resources. (b) Internal innovation material resources. (c) External innovation technology absorption. (d) External innovation technology acquisition. (e) Trade freedom. (f) Financial development. (g) Data application. (h) Data integration.

**Table 1:** Multidimensional innovation factor allocation indicator.

	Dimension	Target layer	Operation layer	Data sources	Processing method
Inputs	Internal innovation factor	Internal innovation human resources	The full-time equivalent of R&D personnel	China Statistical Yearbook on Science and Technology	—
		Internal innovation financial resources	Internal R&D expenditures	China Statistical Yearbook on Science and Technology	Price adjustment and stock adjustment
		Internal innovation material resources	The number of R&D organizations	China Statistical Yearbook on Science and Technology	—
	External innovation factors	External innovation technology cooperation	External R&D expenditures	China Statistical Yearbook on Science and Technology	Price adjustment and stock adjustment
		External innovation technology absorption	Foreign direct investment	China Statistical Yearbook	Exchange rate adjustment, price adjustment, and stock adjustment
		External innovation technology acquisition	High-tech product imports	China Statistical Yearbook on Science and Technology	Exchange rate adjustment and price adjustment
	Institution innovation factors	Property rights protection	The total number of patent enforcement cases	China Statistical Yearbook	—
		Education support	Financial education subsidies	China Statistical Yearbook	Price adjustment
		Trade freedom	Total regional goods exports	China Statistical Yearbook	Exchange rate adjustment and price adjustment
		Trading market	Technology market turnover	China Statistical Yearbook	Price adjustment
		Financial development	Deposits and loans of financial institutions	China Statistical Yearbook	Price adjustment
		Pollution control	Industrial pollution control investment	China Statistical Yearbook	Price adjustment
	Data innovation factors	Data generation	The number of Internet pages	China Statistical Yearbook	—
		Data transmission	Internet broadband access ports	China Statistical Yearbook	—
		Data use	Internet users	China Internet Development Report and China Statistical Yearbook	—
		Data application	Total software services	China Information Yearbook	Price adjustment
		Data sharing	Total post and telecommunications services	China Statistical Yearbook	Price adjustment
		Data integration	The number of robots owned	International Federation of Robotics	Price adjustment
Output		Innovation output	Per capita sales income of new products	China Statistical Yearbook on Science and Technology	Price adjustment

Note: all the data are processed logarithmically to eliminate the influence of differences in indicator units.

**Table 2:** Importance of innovation factor inputs.

Innovation factor inputs	2009	2010	2011	2012	2013	2014	2015	2016	2017	2018	Mean	Ranking
Internal innovation human resources	0.0698	0.0543	0.0693	0.0742	0.0669	0.0579	0.0678	0.0706	0.0639	0.0961	0.0691	7
Internal innovation financial resources	0.0519	0.0530	0.0471	0.0523	0.0368	0.0567	0.0505	0.0600	0.0575	0.0588	0.0525	9
Internal innovation material resources	0.0878	0.0704	0.0636	0.0710	0.0831	0.0894	0.1036	0.1174	0.1105	0.0697	0.0867	4
External innovation technology cooperation	0.0384	0.0455	0.0463	0.0409	0.0502	0.0511	0.0518	0.0453	0.0376	0.0560	0.0463	11
External innovation technology absorption	0.0636	0.0873	0.0833	0.0912	0.1010	0.0824	0.0917	0.0928	0.1064	0.1367	0.0936	3
External innovation technology acquisition	0.0627	0.1031	0.0888	0.0842	0.0742	0.0786	0.0583	0.0616	0.0792	0.0723	0.0763	5
Property rights protection	0.0314	0.0124	0.0173	0.0275	0.0228	0.0235	0.0205	0.0163	0.0158	0.0197	0.0207	16
Education support	0.0183	0.0187	0.0127	0.0132	0.0145	0.0143	0.0146	0.0130	0.0142	0.0149	0.0148	18
Trade freedom	0.0625	0.0560	0.0598	0.0754	0.0766	0.0595	0.0625	0.0682	0.0547	0.0661	0.0641	8
Trading market	0.0692	0.0926	0.0613	0.0241	0.0256	0.0216	0.0198	0.0292	0.0270	0.0294	0.0400	12
Financial development	0.0551	0.0540	0.0623	0.0657	0.0957	0.0837	0.0717	0.0623	0.0787	0.1123	0.0742	6
Pollution control	0.0188	0.0112	0.0156	0.0195	0.0204	0.0094	0.0153	0.0158	0.0267	0.0275	0.0180	17
Data generation	0.0439	0.0391	0.0569	0.0491	0.0627	0.0589	0.0680	0.0386	0.0305	0.0378	0.0485	10
Data transmission	0.0592	0.0338	0.0367	0.0320	0.0439	0.0367	0.0334	0.0227	0.0320	0.0217	0.0352	13
Data use	0.0287	0.0190	0.0201	0.0278	0.0276	0.0250	0.0192	0.0175	0.0182	0.0165	0.0220	15
Data application	0.1078	0.1226	0.1138	0.1008	0.0707	0.0933	0.0876	0.0924	0.0883	0.0653	0.0943	2
Data sharing	0.0294	0.0245	0.0301	0.0301	0.0383	0.0350	0.0324	0.0374	0.0223	0.0215	0.0301	14
Data integration	0.1015	0.1025	0.1150	0.1211	0.0889	0.1227	0.1313	0.1387	0.1367	0.0777	0.1136	1

Note: the ranking results are based on the annual average value.

**Table 3:** Key boundary point of the important innovation factor inputs' marginal effect.

	2009			2012			2015			2018		
	*α*	*β*	*γ*	*α*	*β*	*γ*	*α*	*β*	*γ*	*α*	*β*	*γ*
(a)	7.57	9.39	11.11	7.49	7.50	11.45	7.57	7.58	11.96	9.65	10.28	10.80
(b)	5.70	5.81	7.44	4.34	7.06	7.38	4.44	6.29	8.22	6.17	6.33	8.42
(c)	15.54	18.78	19.20	15.68	19.03	20.24	16.07	19.24	20.38	16.79	18.86	20.97
(d)	11.25	15.21	16.92	9.75	9.76	17.16	9.31	16.35	17.11	12.90	14.42	17.25
(e)	14.02	16.32	17.99	12.88	16.77	18.24	12.15	16.00	18.31	13.36	18.22	18.83
(f)	18.58	18.64	20.38	17.87	17.88	20.80	18.25	19.88	21.31	19.61	20.00	21.51
(g)	12.83	13.51	16.17	9.35	14.36	17.11	10.35	14.19	17.21	14.38	14.54	18.23
(h)	13.99	15.61	16.96	13.20	16.56	17.95	14.42	17.59	19.48	15.50	18.44	20.26

Note: *α, β, γ*, respectively, represent the first turning point, the maximum slope point, and the second turning point boundary value.

**Table 4:** Important innovation factor inputs grouping.

		(a)	(b)	(c)	(d)	(e)	(f)	(g)	(h)
Beijing	2012	4	3	3	3	2	3	4	3
	2018	4	3	3	3	2	3	3	3

Tianjin	2012	3	2	3	3	3	3	3	3
	2018	3	3	3	3	2	3	3	3

Hebei	2012	3	2	2	3	2	3	2	3
	2018	3	3	3	2	2	3	3	3

Shanxi	2012	3	2	2	3	2	3	2	2
	2018	2	1	2	3	2	3	1	2

Inner Mongolia	2012	3	2	2	3	2	3	2	2
	2018	1	1	2	1	2	2	1	2

Liaoning	2012	3	2	3	3	3	3	3	3
	2018	3	3	3	3	2	3	3	2

Jilin	2012	3	2	2	3	2	3	3	3
	2018	2	2	2	2	2	2	3	3

Heilongjiang	2012	3	2	2	3	2	3	2	2
	2018	2	1	2	1	2	2	1	2

Shanghai	2012	3	3	4	4	4	3	3	3
	2018	4	3	4	4	3	3	3	3

Jiangsu	2012	4	4	4	4	4	4	4	4
	2018	4	4	4	4	4	3	3	4

Zhejiang	2012	3	4	3	3	4	4	3	3
	2018	4	3	3	3	3	3	3	3

Anhui	2012	3	2	2	3	2	3	2	3
	2018	3	3	3	3	2	3	3	3

Fujian	2012	3	2	3	3	3	3	3	3
	2018	4	3	3	3	2	3	3	3

Jiangxi	2012	3	2	2	3	2	3	2	2
	2018	3	3	3	3	2	3	1	3

Shandong	2012	3	4	3	3	3	3	3	4
	2018	4	3	3	3	2	3	3	3

Henan	2012	3	2	2	3	2	3	2	3
	2018	3	3	3	3	2	3	3	3

Hubei	2012	3	2	2	3	2	3	3	3
	2018	4	3	3	3	2	3	3	3

Hunan	2012	3	2	2	3	2	3	3	3
	2018	3	3	3	3	2	3	3	3

Guangdong	2012	4	4	4	4	4	4	4	4
	2018	4	4	4	4	4	4	4	4

Guangxi	2012	3	2	2	3	2	3	2	2
	2018	2	2	2	3	2	2	1	2

Hainan	2012	3	2	2	3	2	3	2	2
	2018	1	1	2	2	2	1	2	1

Chongqing	2012	3	2	2	3	2	3	3	3
	2018	3	3	3	3	2	3	3	3

Sichuan	2012	3	2	2	3	2	3	3	3
	2018	4	3	3	3	2	3	3	3

Guizhou	2012	3	2	2	3	2	3	2	2
	2018	1	3	2	2	2	2	1	2

Yunnan	2012	3	2	2	3	2	3	2	2
	2018	2	1	2	2	2	2	1	2

Shaanxi	2012	3	2	2	3	2	3	3	2
	2018	4	3	2	3	2	3	3	2

Gansu	2012	3	2	2	3	2	3	2	2
	2018	1	1	2	1	2	1	1	2

Qinghai	2012	1	1	1	1	1	1	1	1
	2018	1	1	1	1	1	1	1	1

Ningxia	2012	3	1	2	3	2	3	2	2
	2018	1	1	2	1	2	1	1	2

Xinjiang	2012	3	2	2	3	2	3	2	2
	2018	1	1	2	1	2	1	1	2

Note: the input of important innovation factors is divided into group 1 before the first turning point, into group 2 between the first turning point and the maximum slope point, into group 3 between the maximum slope point and the second turning point, and into group 4 after the second turning point.

**Table 5:** Grouping characteristics of important innovation factor inputs.

Grouping characteristics	2012	2018
(a) Part of important innovation factor inputs has not yet reached the starting point of increasing marginal effect	Qinghai, Ningxia	Shanxi, Inner Mongolia, Heilongjiang, Jiangxi, Guangxi, Hainan, Guizhou, Yunnan, Gansu, Qinghai, Ningxia, Xinjiang
(b) All the important innovation factor inputs are in the marginal effects from increasing to maximum and then to falling flat stage	Tianjin, Hebei, Shanxi, Inner Mongolia, Liaoning, Jilin, Heilongjiang, Anhui, Fujian, Jiangxi, Henan, Hubei, Hunan, Guangxi, Hainan, Chongqing, Sichuan, Guizhou, Yunnan, Shaanxi, Gansu, Xinjiang	Tianjin, Hebei, Liaoning, Jilin, Anhui, Henan, Hunan, Chongqing
(c) Part of important innovation factors has completed the input required for the optimal combination of innovation factors	Beijing, Shanghai, Zhejiang, Shandong	Beijing, Shanghai, Jiangsu, Zhejiang, Fujian, Shandong, Hubei, Sichuan, Shaanxi
(d) All the important innovation factor inputs meet the requirements of optimal combination	Jiangsu, Guangdong	Guangdong

## Data Availability

This paper is based on the panel data of 30 provinces in China from 2009 to 2018 (except Tibet). The data sources and processing methods are shown in Table 1.
